The article "Safety Evaluation and Effect Deconstruction of Blood Lipid Test in the Diagnosis of Cardiovascular Disease Patients" was retracted in 2023. Reasons: signs of a paper mill; compromised peer review; unreliable results or conclusions.

# Safety Evaluation and Effect Deconstruction of Blood Lipid Test in the Diagnosis of Cardiovascular Disease Patients

**DOI:** 10.1155/2022/7126659

**Published:** 2022-11-16

**Authors:** Xiaochun Yang, Zhen Lu

**Affiliations:** ^1^Shaoyang University Affiliated Second Hospital, Clinical Laboratory, Shaoyang, 422000 Hunan, China; ^2^Affiliated Hospital of Xiangnan College, Cardiovascular Medicine, Chenzhou, 423000 Hunan, China

## Abstract

With the increase in the number of cardiovascular patients in China, this paper must use better detection methods to examine these patients. Blood lipid testing is a quantitative method for the determination of lipids contained in blood (plasma). Blood lipids are the general term for neutral fats (triglycerides and cholesterol) and lipids (phospholipids, glycolipids, sterols, and steroids) in plasma, which are widely present in the human body. At the same time, this paper also applies this technology to different examination procedures at various current stages. Cardiovascular disease, also known as circulatory system disease, is a series of diseases involving the circulatory system. The circulatory system refers to the organs and tissues that transport blood in the human body, mainly including the heart and blood vessels (arteries, veins, and microvessels), which can be subdivided into acute and chronic and are generally related to arteriosclerosis. In recent years, the most widely used is blood lipid measurement. Therefore, this paper proposes a study on the safety evaluation and effect analysis of blood lipid testing in the diagnosis of cardiovascular disease patients. This article focuses on the causes of cardiovascular disease and introduces the purpose, methods, results, and conclusions of blood lipid detection. Combined with the deep learning method combined with wavelet analysis and support vector machine (SVM), the in-depth analysis is carried out, and suitable patients are selected for blood lipid detection. The final experimental results showed that apolipoprotein B (APOB), total cholesterol (TC), low-density lipoprotein cholesterol (LDL-C), triglyceride (TG), and other indicators were significantly different from the control group. The values of apolipoprotein A1 (APOA1) and high-density lipoprotein cholesterol (HDL-C) were significantly different from those in the control group, *P* < 0.05. This shows that blood lipid examination has a good effect on the diagnosis of cardiovascular patients; it can make accurate diagnosis and prediction of the patient's condition and has good clinical application value.

## 1. Introduction

The clinical incidence of cardiovascular disease is increasing day by day, posing a serious threat to human health. In particular, in developing countries, the death toll accounts for about 40%. Cardiovascular disease is a common disease among middle-aged and elderly people. The cardiovascular system is irreplaceable in the process of maintaining the physiological needs of the human body. Once the system is disturbed, the entire physiological function will be affected. With the advancement of medical technology, the diagnosis and treatment of cardiovascular disease should comprehensively consider the patient's condition, type, and severity. Early symptoms are atypical and difficult to diagnose. In order to make accurate predictions of patients' diseases as early as possible, people are always looking for an effective method for disease diagnosis and prediction. The blood lipid detection technology is the best method at present, which can detect and prevent its occurrence in time. At present, it is clinically recognized that blood lipid changes are related to cardiovascular disease, and more and more attention has been paid to blood lipid testing for the diagnosis of cardiovascular disease.

The article "Safety Evaluation and Effect Deconstruction of Blood Lipid Test in the Diagnosis of Cardiovascular Disease Patients" was retracted in 2023. Reasons: signs of a paper mill; compromised peer review; unreliable results or conclusions.

This paper mainly introduces the causes of cardiovascular disease and its electrocardiographic signal processing technology and uses the wavelet transform and support vector machine theory in the deep learning algorithm to perform in-depth analysis and calculation. Then, select appropriate patients for testing to test blood lipids. The innovation of this article is that the article uses multiple experiments for analysis. Moreover, the deep learning is also analyzed in detail in the algorithm part, and it is used in the treatment of cardiovascular diseases, which is very practical, so the experimental data and conclusions are more accurate and have more medical value.

## 2. Related Work

With the accelerated pace of China's entry into an aging society, there are more and more elderly people in China, which means that cardiovascular disease has gradually become a concern of the whole society. The work of cardiovascular medicine nurses also puts forward higher requirements, and the content of traditional nursing work has more profound changes. The development of medical technology has made patients experience the end of their lives. As life grows, so does the life of the disabled. In old age, heart disease patients are especially prone to it. Wang analyzed the subjects' physiological parameters such as blood sugar and blood lipids and used Illumina high-throughput sequencing technology to analyze their fecal microbiota [1]. Modern medicine also brings new ethical challenges. Warraich made some recommendations for improving end-of-life care services for cardiovascular patients, such as optimizing assessment quality indicators, closing gaps, strengthening education and research, overcoming gaps, and providing and complementing palliative care [2]. Nielsen presented the short-term and long-term cardiovascular effects of mediastinal radiation therapy and evaluated asymptomatic and symptomatic patients [3]. The goal of Ozkan et al. is to measure the risk of cardiovascular disease [4]. Although their articles all studied the conditions of patients with cardiovascular disease and their treatment methods, they did not conduct in-depth research on their blood lipid detection methods, nor did they use deep learning algorithms for optimization.

The article "Safety Evaluation and Effect Deconstruction of Blood Lipid Test in the Diagnosis of Cardiovascular Disease Patients" was retracted in 2023. Reasons: signs of a paper mill; compromised peer review; unreliable results or conclusions.

Dong and Li mainly studied acoustic models based on deep learning [5]. Oshea brought new deep learning applications to the physical level. The communication technology was regarded as a basic coding method, and the design of the communication system is regarded as a point-to-point combination so that the transmission and reception links can be optimally solved [6]. Because technology is still so low, a system that can automatically identify diseases could save lives, reduce unnecessary biopsies, and reduce costs. To achieve this, Codella et al. had developed a new system that combined deep learning with machine learning [7]. They all introduced the basic situation of deep learning network and its algorithm research, but the application in cardiovascular disease has not been introduced in detail, so it still does not have enough influence on medicine [8].

## 3. Cardiovascular Disease Algorithm under Deep Learning

### 3.1. ECG Signal Preprocessing Technology

#### 3.1.1. The Mechanism of ECG Signal Generation

The heart is a major organ in the circulatory system of higher animals. The main function is to provide pressure for blood flow and to run the blood to all parts of the body. The heart is like an energy source that transmits all motor potentials to the surface of the body. Some individual surfaces have larger potential differences, while others have larger potential differences. The motion of the heart is determined by the electrophysiological phenomena of cardiomyocytes—depolarization and repolarization. The heart and its structure are shown in Figure 1 [9, 10].

As shown in Figure 2, cardiomyocytes are short columnar and generally have only one nucleus, while skeletal muscle fibers are multinucleated cells. There are intercalated disc structures between cardiomyocytes. The myocardial cell membrane is essentially a semipermeable membrane. At rest, a certain amount of positively charged cations is arranged on the semipermeable membrane, and the negative potential inside the semipermeable membrane is lower than that outside the membrane, that is, polarization [11, 12]. In each cardiac cycle, the heart is excited successively by the pacemaker, atrium, and ventricle. Along with the changes of bioelectricity, various patterns of potential changes are drawn from the body surface through the electrocardiograph. When not moving, the cardiomyocytes in various parts of the heart are polarized, with no potential difference, and the current recorder draws a line, the body's electrocardiogram. Under the action of the semipermeable membrane, the permeability of cells to potassium, chloride, sodium, and calcium ions changes, resulting in depolarization and repolarization of cardiomyocytes. And it forms a pair of galvanic couples with the cell membrane of adjacent cells, resulting in a change in potential.

The article "Safety Evaluation and Effect Deconstruction of Blood Lipid Test in the Diagnosis of Cardiovascular Disease Patients" was retracted in 2023. Reasons: signs of a paper mill; compromised peer review; unreliable results or conclusions.

#### 3.1.2. Wavelet Transform

If its Fourier transform satisfies the condition [13, 14]

(1) $$\begin{array}{c} \beta \left(d\right)=\overset{K}{\int \frac{\left|\beta {\left(\varepsilon \right)}^{2}\right|}{\varepsilon }}t\varepsilon <\infty , \end{array}$$

then

(2) $$\begin{array}{c} \beta_{\chi ,\alpha }\left(d\right)=\chi^{1/2}\beta \left(\frac{d-\alpha }{\chi }\right),\;\chi >0,\;\alpha \in K. \end{array}$$

Its expression is

(3) $$\begin{array}{c} {SD}_{g}\left(\chi ,\alpha \right)\leq g\left(d\right),\\ \beta_{\chi ,\alpha }\left(d\right)\geq \frac{1}{\sqrt{\chi }}\overset{K}{\int g\left(d\right)\beta \left(\frac{d-\alpha }{\chi }\right)td}. \end{array}$$

According to this Marat algorithm, the decomposition of its orthogonal wavelet transform is

(4) $$\begin{array}{c} e_{i,r}=\underset{m}{\sum }e_{i-1,m}g_{m-2r},\\ t_{i,r}=\overset{m}{\underset{m}{\sum }}t_{i-1,m}g_{m-2r}. \end{array}$$

The wavelet transform reconstruction process of the discrete signal is as follows:

(5) $$\begin{array}{c} e_{i-1,m}=\underset{m}{\sum }e_{i,m}g_{r-2m}+\underset{m}{\sum }t_{i,m}g_{r-2m}. \end{array}$$

This transform is called a second-order wavelet transform and has basis functions:

(6) $$\begin{array}{c} \beta_{r,z}\left(d\right)=2^{-r/2}\beta \left(2^{-r}d-z\right),\;r,z\in L^{+}. \end{array}$$

From the concept of space, the multiresolution characteristics of wavelets are vividly illustrated. As the scale changes from large to small, it is an algorithm that can observe different characteristics of the image from coarse to fine at each scale.

#### 3.1.3. Support Vector Machine

The so-called support vector refers to those training sample points on the edge of the interval. The “machine” here is actually an algorithm. In the field of machine learning, some algorithms are often regarded as a machine.

For *mn*-dimensional linear inseparable samples

(7) $$\begin{array}{c} \left(a_{1},b_{1}\right),\cdots \left(a_{m},b_{m}\right)\in K^{n}\times \left\{-1,1\right\},\\ b_{j}\left[\varepsilon *\beta \left(a_{j}\right)+y\right]\geq 1,\;j=1,2,\cdots m,\\ \min I\left(\varepsilon ,\gamma \right)=\frac{1}{2}\left\|\varepsilon \right\|+E\overset{n}{\underset{j=1}{\sum }}\gamma_{j},\\ \text{w}.\text{d}.b_{j}\left[\varepsilon *\beta \left(a_{j}\right)+y\right]\geq 1-\gamma_{j},\;\gamma_{j}\geq 0,\;j=1,2,\cdots M,\\ g\left(a\right)=\mathrm{sgn}\left[\overset{1}{\underset{j=1}{\sum }}\chi_{j}b_{j}R\left(a,a_{j}\right)+y\right]. \end{array}$$

The article "Safety Evaluation and Effect Deconstruction of Blood Lipid Test in the Diagnosis of Cardiovascular Disease Patients" was retracted in 2023. Reasons: signs of a paper mill; compromised peer review; unreliable results or conclusions.

#### 3.1.4. Deep Residual Network

Deep convolutional neural networks have led to a series of breakthroughs in image classification. By varying the number of layers (depth), deep networks naturally integrate low/medium/high level features, layers in an end-to-end multilayer fashion, and feature “levels” all become richer. However, deeper networks suffer from gradient dispersion problems during backpropagation [15, 16]. The reason for the low performance of gradient descent on deep networks with randomly initialized weights is that the gradient gets smaller and smaller during backpropagation [17, 18]. Specifically, a simple neural network can be set up, as shown in Figure 3 [19].

From the basic working principle of the convolutional neural network, the update formula of *b*_1_ can be deduced as

(8) $$\begin{array}{c} b_{1}=b_{1}-\chi \frac{tB}{{tb}_{1}}. \end{array}$$

Among them,

(9) $$\begin{array}{c} \frac{tB}{{tb}_{1}}=g^{\prime }\left(l_{1}\right)\times a_{2}\times g^{\prime }\left(l_{2}\right)\times a_{3}\times g^{\prime }\left(l_{3}\right)\times a_{4}\times g^{\prime }\left(l_{4}\right)\times \frac{tB}{{tu}_{4}}. \end{array}$$

*u*_4_ represents the output generated by the fourth convolutional layer of the neural network.

Its structure is shown in Figure 4.

#### 3.1.5. Long Short-Term Memory Network (LSTM)

As shown in Figure 5, it performs the same operation for every element in the sequence. Each operation relies on the results of previous computations, processing the entire sequence in such a way that the final hidden state contains information from all its previous elements.

There is loss of information due to the decay of gradient values over time during backward propagation. The gradient calculation formula of RNN hidden layer 14 is

(10) $$\begin{array}{c} \eta_{g}^{d}=\frac{\phi }{\phi x_{g}^{d}}=\varphi^{\prime }\left(x_{g}^{d}\right)\left(\overset{G}{\underset{g^{\prime }=1}{\sum }}\eta_{g^{\prime }}^{d+1}s_{gg^{\prime }}\right). \end{array}$$

And this paper assumes that only the hidden layer of the last moment *D* has output, so there is a simplification of the formula; let *d* = 1, then

(11) $$\begin{array}{c} \eta_{g_{1}}^{1}=\varphi_{g}^{\prime }\left(x_{g_{1}}^{1}\right)\left(\overset{G}{\underset{g_{2}}{\sum }}\eta_{g_{2}}^{2}s_{g_{1}g_{2}}\right). \end{array}$$

Of course, there are also more general forms as follows:

(12) $$\begin{array}{c} \eta_{g_{1}}^{d}=\overset{G}{\underset{g_{d+1=1}}{\sum }}\cdots \overset{G}{\underset{g_{D}=1}{\sum }}\overset{G}{\underset{r=1}{\sum }}\left(b_{r}^{D}-l_{r}^{D}\right)s_{g_{D}r}\overset{D-1}{\underset{n=1}{\prod }}\phi_{g}^{\prime }\left(x_{g_{n}}^{n}\right)s_{g_{n}g_{n+1}}. \end{array}$$

It can be seen that the right side of the formula is equivalent to having *D* consecutive multiplications in the form of *φ*′*s*; then, when *D* is larger, the following two situations will occur:

(13) $$\begin{array}{c} \left\{\begin{array}{c} \eta_{g}^{d}⟶\infty \text{if}\left|\varphi^{\prime }s\right|>1.0\\ \eta_{g}^{d}⟶0\text{ if}\left|\varphi^{\prime }s\right|<1.0 \end{array}\right\}. \end{array}$$

Long short-term memory network is a temporal recurrent neural network suitable for processing and predicting important events with relatively long intervals and delays in time series. Long short-term memory networks introduce a constraint that solves this problem by using more complex hidden layer node activations to preserve long-term state information.

The article "Safety Evaluation and Effect Deconstruction of Blood Lipid Test in the Diagnosis of Cardiovascular Disease Patients" was retracted in 2023. Reasons: signs of a paper mill; compromised peer review; unreliable results or conclusions.

The long short-term memory network replaces each hidden layer node with the memory block shown in Figure 6.

(14) $$\begin{array}{c} j_{d}≔\text{sigmoid}\left[S_{gj}*g_{d-1}+S_{aj}*a_{d}+y_{j}\right]. \end{array}$$

### 3.2. Standard ECG Database

Table 1 shows the sampling distribution of ECG signals.

As shown in Table 2, due to the fact that some ECG examples in the real clinical environment have some lead-off, abnormal QRS waveforms, invalid records, etc., some examples are invalid.

This paper uses a ratio of about 70 : 30 to divide the dataset, that is, about 70% of the dataset used for training and about 30% of the dataset used for network testing. This is the standard ratio for dividing datasets in machine learning datasets. The advantage of this partitioning is that it provides enough data for training and testing the system, avoiding deficiencies that can occur when the training dataset is smaller than the testing dataset. Also, if the training dataset is much larger than the test dataset, it may cause the system to overfit.

## 4. Application of Blood Lipid Test in Patients with Cardiovascular Disease

### 4.1. Sample Error Test

This article conducted an interview with a hospital during the treatment. During these two years, the hospital admitted an average of 60 patients with diabetes, of which 45 were men, with an average age of 62, while there are only 15 women and the average age is only 53 years old. The World Health Organization (WHO) is a specialized agency under the United Nations. Its headquarters is located in Geneva, Switzerland, and only sovereign states can participate. It is the largest intergovernmental health organization in the world, with 194 member states as of 2015. The specific conditions of the patients are shown in Figure 7, and a variety of tests have been performed on these patients in accordance with the relevant regulations of the World Health Organization (WHO). During hospitalization, they experience coma, dizziness, fatigue, chest pain, and elevated triglyceride levels.

The article "Safety Evaluation and Effect Deconstruction of Blood Lipid Test in the Diagnosis of Cardiovascular Disease Patients" was retracted in 2023. Reasons: signs of a paper mill; compromised peer review; unreliable results or conclusions.

The laboratory is a very important department. On the whole, the laboratory is responsible for the detection of immunization, microbiology, clinical inspection, and biochemistry. Blood test is an important part of clinical examination and an important technique for clinical diagnosis and analysis of the disease [20]. Its accuracy is closely related to clinical diagnosis and treatment; therefore, it is particularly important to improve the accuracy of test results.

As shown in Figure 8, there are many types of sample errors in blood tests. 32 samples caused errors during the inspection process, accounting for 40% of the total errors. And 16 samples were due to collection, accounting for 20% of the total error; 14 samples were caused by hemolysis, accounting for 17.5% of the total error. 10 samples were caused by nonstandard testing, accounting for 12.5% of the total error, and 8 samples were caused by the patient's own factors, accounting for 10% of the total error.

The following methods can be adopted in this paper. First, reduce the blood sugar concentration of the patient and reduce the sensitivity to insulin. At the same time, the stability of elements in the body can also be achieved by adjusting the content of esters and reducing the content of esters. In addition, specific receptor-blocking drugs can be used to reduce sudden death in people with diabetes.

### 4.2. Blood Lipid Test Can Be Helpful to the Disease Process of Patients

The two groups of patients took 5 mL of venous blood on an empty stomach in the morning, soaked in water bath for 30 minutes after 30 minutes, centrifuged at 3000 r/min, and separated plasma after 10 minutes. Plasma samples were placed in an anticoagulation catheter, and their blood lipids, including APOA1, HDL-C, TC, APOB, LDL-C, and TG, were detected by a blood biochemical analyzer. The detection of HDL-C, TC, and TG is carried out by enzymatic method, that is, the use of lipid reagents, and the corresponding detection is carried out according to the instructions.

The article "Safety Evaluation and Effect Deconstruction of Blood Lipid Test in the Diagnosis of Cardiovascular Disease Patients" was retracted in 2023. Reasons: signs of a paper mill; compromised peer review; unreliable results or conclusions.

Observation indicators: APOB, TC, LDL-C, TG, APOAI, HDL-C, and other indicators were compared. The normal values of all indicators are as follows: low-density lipoprotein cholesterol 2.08-3.02 mmol/L; HDL-C 1.61 mmoL/L-1.66 mmoL/L; TC is 3.1 mmoL/L-5.7 mmoL/L; TG is 0.35 mmoL/L-1.71 mmol/L.

The results showed that APOB, TC, LDL-C, TG, and other indicators were significantly decreased compared with normal people; APOAI and HDL-C were significantly lower than the control group, *P* < 0.05; see Figure 9 for details.

Cardiovascular disease is clinically a disease with high mortality and high disability and is the main cause of harm to human health. Although the treatment of this disease is more difficult, if it can be detected and prevented early, the quality of life of the patient can be improved. At the time of diagnosis, blood lipid testing can be used to understand the condition, help doctors formulate treatment plans, and improve the prognosis of patients. At present, blood lipid detection mainly uses APOAI, HDL-C, TC, APOB, LDL-C, TG, and other indicators and compares them with normal values to determine the risk of the disease.

The results showed that APOB, TC, LDL-C, TG, and other indicators were significantly higher than those of the control group, and the values of APOAI and HDL-C were significantly different from those of the control group, *P* < 0.05. Therefore, adults and patients should regularly go to the hospital for blood lipid testing in order to detect and treat in time, improve prognosis, and prevent further deterioration of the disease. Therefore, blood lipid detection has a certain guiding role in the diagnosis of cardiovascular disease [21]. In conclusion, blood lipid detection has a good effect on the diagnosis of cardiovascular patients. It can make an accurate diagnosis of the patient's condition, can make an accurate prediction of the patient's condition, and has good clinical application value.

### 4.3. Clinical Value of Blood Lipid Test in the Diagnosis of Patients with Cardiovascular Disease

Taking 80 cases of the experimental group and the control group as the research objects, the role of blood lipid detection in cardiovascular diseases was studied. As shown in Table 3, there were 20 male patients and 20 female patients, 33-63 years old, with an average age of 54.39 ± 2.47. The control group consisted of 20 cases, ranging from 34 to 65 years old, with an average age of 53.98 ± 3.21. All patients expressed their informed consent to this study, and the overall data was compared (*P* > 0.05), which was confirmed by the hospital ethics committee.

The article "Safety Evaluation and Effect Deconstruction of Blood Lipid Test in the Diagnosis of Cardiovascular Disease Patients" was retracted in 2023. Reasons: signs of a paper mill; compromised peer review; unreliable results or conclusions.

Both groups underwent routine blood lipid testing. Mindray automatic biochemical analyzer was used to determine serum TC, HDL-G, LDL-C, and serum triacylglycerol (TG). At the same time, 2 mL of venous blood was randomly drawn, and the plasma concentration, erythrocyte aggregation, and erythrocyte deformability were measured by Beijing Pulisheng automatic rheometer.

Results: compared with the control group, the blood rheology indexes of the two groups of patients are shown in Table 4. The results showed that the aggregation rates of plasma and erythrocytes in the two groups of patients were higher than those of normal subjects, while the degree of degeneration of erythrocytes was significantly different.

The blood lipid indexes of each group and the control group were observed and compared. The results showed that compared with the control group, the HDL-G level in the experimental group was significantly lower, and the LDL-C, TC, and TG values were significantly higher than those in the control group as shown in Figure 10.

Blood lipids play a major role in cardiovascular disease. Four items of total cholesterol, LDL cholesterol, low-density lipoprotein cholesterol, and serum triacylglycerol are tested for blood lipids. If the serum triacylglycerol monoindex increases and the high-density lipoprotein cholesterol level decreases, it is cardiovascular disease.

Lipid testing is a method of quantifying the amount of fat in the body. The detection of blood lipids includes total cholesterol, triglycerides, high-density lipoprotein, and low-density lipoprotein. Therefore, patients with family history of cardiovascular disease, hypertension, coronary heart disease, etc., if there are patients with cardiovascular disease, blood lipid testing must be carried out regularly. Therefore, blood lipid detection is an effective auxiliary means. For patients with cardiovascular disease, in addition to blood lipid testing, their blood rheology indicators are also higher than those of the normal population. At the same time, the hemorheology index is also an important index of cardiovascular disease.

In general, the blood lipid indicators of patients with cardiovascular disease are far from those of normal people. Therefore, regular monitoring of blood lipids, combined with hemorheological indicators, early diagnosis, and early treatment can avoid the aggravation of the disease and improve the prognosis [22].

## 5. Conclusions

From the research and analysis of the above cases, it can be seen that in China's current medical level, diabetes and cardiomyopathy are very difficult to diagnose and treat. Moreover, the etiology is also very complex, and the etiology and treatment methods of the disease must be analyzed in detail according to different cases and experiences. At the same time, this article also needs to continuously update the therapy and treatment plan of this article so that this disease can be better controlled. As a common clinical examination method, blood lipid detection is of great significance for the prediction, early diagnosis, and early treatment of cardiovascular disease. In addition, after the clinical diagnosis of cardiovascular disease, it is necessary to propose effective treatment measures in time, adjust the patient's psychological state, and allow the patient to receive treatment in the best psychological state, encouraging the patient to strengthen physical exercise and enhance physical immunity. In conclusion, early diagnosis of cardiovascular disease based on blood lipid test can accurately assess the degree of cardiovascular disease, which has important reference significance for the subsequent clinical diagnosis of cardiovascular disease.

The article "Safety Evaluation and Effect Deconstruction of Blood Lipid Test in the Diagnosis of Cardiovascular Disease Patients" was retracted in 2023. Reasons: signs of a paper mill; compromised peer review; unreliable results or conclusions.

## Figures and Tables

**Figure 1:** The heart and its structure.

**Figure 2:** ECG signal processing technology.

**Figure 3:** Common convolutional neural network.

**Figure 4:** Residual learning: a shortcut link structure.

**Figure 5:** Symbolic representation of recurrent neural network (RNN) and equivalent extensions.

**Figure 6:** Structure figure of the core cell of the long short-term memory network.

**Figure 7:** Statistical figure of patient status.

**Figure 8:** Analysis of factors for the occurrence of errors in blood samples.

**Figure 9:** Comparison of test results between the two groups.

**Figure 10:** Comparison of blood lipid levels in the two groups of patients.

**Table 1:** Sample distribution of all sample datasets and positive abnormal ECG signals.

	Normal (0)	Normal (1)
Train set	136110	6327
Train set A	6808	3163
Train set B	54470	25309
Sun	74890	34800

**Table 2:** Data distribution of the dataset.

Data serial number	Normal	Abnormal	Total
1	17467	7202	24667
2	4911	6352	11263
3	25020	19249	35269
4	16210	6508	22718
5	10351	12948	23299
6	9703	11529	21232

**Table 3:** Detailed statistics of patients in the control group and the study group.

Group	Gender	Number of people	Average age	Age
Research group	Man	20	(54.39 ± 2.47)	33-63
	Woman	20		

Control group	Man	20	(53.98 ± 3.21)	34-65
	Woman	20		

**Table 4:** Comparison of hemorheological indexes between the observation group and the control group.

Group	Number of cases	Plasma concentration	Red blood cell aggregation	RBC deformability
Observation group	40	3.7 ± 1.8	5.9 ± 1.3	0.5 ± 0.7
Control group	40	1.2 ± 0.2	3.7 ± 1.4	1.8 ± 0.9
*T* value	/	11.4	18.2	16.1
*P* value	/	<0.05	<0.05	<0.05

The article "Safety Evaluation and Effect Deconstruction of Blood Lipid Test in the Diagnosis of Cardiovascular Disease Patients" was retracted in 2023. Reasons: signs of a paper mill; compromised peer review; unreliable results or conclusions.

## Data Availability

This article does not cover data research. No data were used to support this study.
